The article "Nomogram for Predicting Deep Venous Thrombosis in Lower Extremity Fractures" was retracted in 2024. Reasons: signs of a paper mill; suspected computer-generated content; unreliable results or conclusions; concerns about the data.

# Nomogram for Predicting Deep Venous Thrombosis in Lower Extremity Fractures

**DOI:** 10.1155/2021/9930524

**Published:** 2021-06-22

**Authors:** Ze Lin, Bobin Mi, Xuehan Liu, Adriana C. Panayi, Yuan Xiong, Hang Xue, Wu Zhou, Faqi Cao, Jing Liu, Liangcong Hu, Yiqiang Hu, Lang Chen, Chenchen Yan, Xudong Xie, Junfei Guo, Zhiyong Hou, Yun Sun, Yingze Zhang, Yu Hu, Guohui Liu

**Affiliations:** ^1^Department of Orthopaedics, Union Hospital, Tongji Medical College, Huazhong University of Science and Technology, Jiefang Road. 1277#, Wuhan, 430022 Hubei, China; ^2^Tongji Medical College, Huazhong University of Science and Technology, Wuhan 430022, China; ^3^The Division of Plastic Surgery, Brigham and Women's Hospital, Harvard Medical School, Boston, MA, USA; ^4^Department of Orthopaedic Surgery, The Third Hospital of Hebei Medical University, No. 139 Ziqiang Road, Shijiazhuang, 050051 Hebei, China; ^5^Key Laboratory of Biomechanics of Hebei Province, Shijiazhuang, 050051 Hebei, China; ^6^Institute of Hematology, Union Hospital, Tongji Medical College, Huazhong University of Science and Technology, Wuhan, 430022 Hubei, China

## Abstract

Deep venous thrombosis (DVT) is a common complication in patients with lower extremity fractures, causing delays in recovery short-term and possible impacts on quality of life long-term. Early prediction and prevention of thrombosis can effectively reduce patient pain while improving outcomes. Although research on the risk factors for thrombosis is prevalent, there is a stark lack of clinical predictive models for DVT occurrence specifically in patients with lower limb fractures. In this study, we aim to propose a new thrombus prediction model for lower extremity fracture patients. Data from 3300 patients with lower limb fractures were collected from Wuhan Union Hospital and Hebei Third Hospital, China. Patients who met our inclusion criteria were divided into a thrombosis and a nonthrombosis group. A multivariate logistic regression analysis was carried out to identify predictors with obvious effects, and the corresponding formulas were used to establish the model. Model performance was evaluated using a discrimination and correction curve. 2662 patients were included in the regression analysis, with 1666 in the thrombosis group and 996 in the nonthrombosis group. Predictive factors included age, Body Mass Index (BMI), fracture-fixation types, energy of impact at the time of injury, blood transfusion during hospitalization, and use of anticoagulant drugs. The discriminative ability of the model was verified using the C-statistic (0.676). For the convenience of clinical use, a score table and nomogram were compiled. Data from two centers were used to establish a novel thrombus prediction model specific for patients with lower limb fractures, with verified predictive ability.

The article "Nomogram for Predicting Deep Venous Thrombosis in Lower Extremity Fractures" was retracted in 2024. Reasons: signs of a paper mill; suspected computer-generated content; unreliable results or conclusions; concerns about the data.

## 1. Introduction

Lower limb fractures account for approximately one-third of fracture patients [1–3], with a higher incidence in the elderly population. Consequently, given the aging population, lower limb fractures are on the rise. Among hospitalized patients, trauma patients have the highest risk of developing deep venous thrombosis (DVT), with the risk reported to be 13-fold higher than nontrauma patients [4, 5].

Further, lower limb fractures are a well-known risk factor for DVT occurrence [6]. DVT is in turn the third leading cause of cardiovascular death worldwide [7, 8] and also a major complication limiting recovery in patients with lower limb fractures [6, 9].

Thrombosis in patients with fractures is primarily formed in the deep veins of the lower extremities, which may result in swelling and pain in the patient's lower extremities. When the thrombus dislodges, it may cause life-threatening complications such as pulmonary embolism [7, 10–12]. A large number of studies have investigated the diagnosis and treatment of DVT. Specific advances include the combination of ultrasound, D-dimer, and clinical evaluation for thrombosis diagnosis [13, 14]; the use of small RNA molecules as new diagnostic markers [15, 16],; and the combination therapy and standard treatment with anticoagulation and antithrombotic drugs [7, 9]. In comparison to the large strides that have been made in the treatment of thrombosis, efforts to increase early prediction and prevention of DVT—which are arguably more effective and more efficient—have been minimal. Therefore, early prediction of thrombosis has become a major focus of current research.

An increasing number of studies have strove to identify the factors associated with DVT occurrence during hospitalization of patients with lower limb fractures [8, 17–19]. Such studies have offered a better understanding of the factors associated with increased DVT risk. However, whether to take the prevention of DVT is usually based on a physician's experience and on patient symptoms. Although practical, this approach may delay the prevention and treatment of DVT. Identification of patients who are at the highest risk of DVT may enable the provision of timely and effective therapies, thereby avoiding DVT occurrence.

Although there are several prediction models for venous thrombosis, like Caprini Risk Assessment Model, these are not specific to lower extremity fractures and, hence, have several limitations if used in that context. First, some tools already used in clinic fail to include factors that may affect thrombosis which are specific to fracture patients, including energy of impact and surgical method. This highlights the need for a more targeted prediction model. Second, some studies focus on the effect of a single risk factor for thrombosis in fracture patients [20, 21]. However, the occurrence of thrombosis is a relatively complicated, multifactorial process [6]. Therefore, the ability of single factor prediction is limited. Furthermore, some studies that do include multiple influencing factors fail to establish a clear clinical predictive model or a scoring table that can be applied by physicians in a healthcare setting [22–24]. In order to be able to translate such research results to patient care, a prediction model must be established. The primary aim of this study is to develop a model for predicting the risk of DVT following a lower limb fracture and, ultimately, offers a straight-to-clinic/hospital nomogram that can change current practice.

The article "Nomogram for Predicting Deep Venous Thrombosis in Lower Extremity Fractures" was retracted in 2024. Reasons: signs of a paper mill; suspected computer-generated content; unreliable results or conclusions; concerns about the data.

## 2. Materials and Methods

### 2.1. Study Population

This retrospective cohort study consisted of two groups (thrombosis group and nonthrombosis group) of patients with lower limb fractures who underwent surgery at Wuhan Union Hospital and Hebei Third Hospital, China. Patients with hip, femur, or tibial fibula fractures were included in the study. At the same time, patients who had experienced a DVT prior to the fracture were excluded from the study. The time frame for the collection of medical records was from January 2016 to January 2019. The information collected consisted of 18 risk factors linked to DVT occurrence in the lower extremities, such as sex, age, site of fracture, history of cardiovascular disease, and BMI. The current study was approved by the Ethics Committee of Union Hospital, Tongji Medical College, Huazhong University of Science and Technology.

### 2.2. Clinical Outcomes and Definitions

The defined outcome was the occurrence of lower extremity DVT. Venous ultrasound is the gold standard for establishing whether DVT has formed in the lower extremities [25, 26]. When the patient's lower extremity venous ultrasound results show that venous thrombosis has formed, the patient was included in the thrombosis group. All lower extremity venous ultrasound findings included in this study were recorded in the patient's medical history data during hospitalization. In patients with femur or tibia/fibula fractures, the venous ultrasound was performed on the noninjured lower extremity. In patients with hip fractures, the test was performed on both lower limbs, and the result of the side with the more severe thrombosis was recorded. Patients who did not undergo a lower limb venous ultrasound examination during hospitalization were excluded from the analysis.

The article "Nomogram for Predicting Deep Venous Thrombosis in Lower Extremity Fractures" was retracted in 2024. Reasons: signs of a paper mill; suspected computer-generated content; unreliable results or conclusions; concerns about the data.

### 2.3. Selection of Predictors

Firstly, we selected the factors that significantly affect the formation of thrombus as potential predictors. A list of potential predictors was compiled from a search of the relevant literature as well as through clinical judgment. These variables were sex, age, BMI, fracture site, energy of the traumatic impact, open wound, traumatic brain injury, cardiovascular history, history of type II diabetes, smoking history, triglyceride (TG), high-density lipoprotein (HDL), low-density lipoprotein (LDL), D-dimer, prothrombin time (PT), activated partial thromboplastin time (APTT), thrombin time (TT), fibrinogen (FIB), duration of surgery, fracture fixation types, blood transfusion during hospitalization (red blood cells), and anticoagulation drugs (low-molecular-weight heparin sodium; Table 1). The fracture sites were divided into hip, femur, and tibia/fibula. Traumatic brain injury was determined through head imaging. Fracture fixation types included internal fixation, external fixation, and others.

### 2.4. Missing Data

In this retrospective study, 19.33% (*n* = 638) of patients had missing medical history information or test results due to the long review period. Participants with missing ultrasound results were also excluded. In the case of participants with missing basic information, a multiple filler method was used to supplement the data.

### 2.5. Model Building

Data analysis of the individual variables was performed using *χ*^2^  or CMH-*χ*^2^, Fisher exact probability test, and Wilcoxon rank-sum test for between-group comparison to identify variables significantly associated with DVT. Risk factors with significant univariate associations (*p* < 0.05) were incorporated into the multivariate model. The regression coefficients *β*, OR, and 95% CI for each risk factor were estimated by constructing a multivariate logistic regression model that incorporated the risk factors primarily considered in the regression model. Nomogram coefficients for each variable were calculated based on coefficients from logistic regression and data according to the formula: Nomogrami = (max(Wi) − min(Wi))∗*β*i. In this formula, max (W) and min (W) represent the maximum and minimum values of each variable. Subsequently, we selected age as the scoring scale, with a total score of 100. After clarifying the score corresponding to age, we calculated the score corresponding to each variable according to the coefficient: Pointi = 100∗(Nomogrami/Nomogramage)/(max(Wi) − min(Wi). In the model testing process, internal validation of the models was conducted using the bootstrap method with 1000 replicates. And we used the c-statistic to measure the discrimination of our model. This study was performed according to the Transparent Reporting of a multivariable prediction model for Individual Prognosis or Diagnosis (TRIPOD) statement.

The article "Nomogram for Predicting Deep Venous Thrombosis in Lower Extremity Fractures" was retracted in 2024. Reasons: signs of a paper mill; suspected computer-generated content; unreliable results or conclusions; concerns about the data.

### 2.6. Sample Size

In this retrospective study, we collected 3300 medical records from two centers. 638 records were not eligible for use in the model building process due to missing data or examination results. The remaining 2662 were included in the clinical prediction model building. According to established criteria for constructing clinical prediction models, this amount of data is adequate for model construction [27].

### 2.7. General Statistical Methods

Model building and nomogram plotting were performed using the rms package in R (version 3.6.1; Windows; R Core Team [28]) through RStudio (version 1.2.5001; R Studio Team [29]).

## 3. Results

### 3.1. Sample Characteristics and Outcomes

Patient characteristics are summarized in Table 1. We collected the medical records of thrombotic patients (*n* = 1666) and nonthrombotic patients (*n* = 996). 2034 patients were diagnosed with femur fractures and 387 patients were diagnosed with tibia/fibula fractures. In the thrombosis group, 870 (52.22%) of the patients were male, the median age was 73 years old, the majority (66.15%) of patients had a history of cardiovascular disease, 1447 (86.85%) patients did not have a history of type II diabetes, and nearly half (47.24%) of the patients had a blood transfusion during their hospitalization. In the nonthrombosis group, median BMI was 23.88, 73 (7.33%) patients had an open wound, most (94.58%) patients did not have a traumatic brain injury, and only a few (4.22%) patients were not treated with anticoagulation drugs. There was no significant difference between the groups in terms of traumatic brain injury occurrence, smoking history, blood lipid levels, TT, FIB, and duration of surgery. Comparisons between the groups for each variable are also shown in Table 1.

### 3.2. Model Development

Multivariate logistic regression analysis was performed on identified potential predictors of thrombosis (*p* < 0.05). After completion of the regression analysis, variables lacking statistical significance were eliminated. Regression coefficients for each predictor in the final prediction model are recorded in Table 2. The predictors included in this thrombosis prediction model were age, BMI, energy of impact, fracture fixation type, blood transfusion during hospitalization, and use of anticoagulation drugs. The c-statistic of this thrombus-related clinical prediction model is 0.676, highlighting the model's good discriminatory ability. During the internal validation of the model, a correction curve was drawn using R (Figure 1). The curve shows that the prediction model has a good fit to the real scenario.

The article "Nomogram for Predicting Deep Venous Thrombosis in Lower Extremity Fractures" was retracted in 2024. Reasons: signs of a paper mill; suspected computer-generated content; unreliable results or conclusions; concerns about the data.

### 3.3. Computing the Risk Estimate and Nomogram Presentation

After completing the multivariate logistic regression analysis, we calculated the nomogram coefficient of age as per the formula defined in the methods (Nomogram_Age_ = 1.728). As we intended to use age as the scoring scale (with a total score of 100), we used 10 years as a baseline reference (i.e., Point_age=10_ = 0) with the total score increasing by 1 for each additional year of age. After completing the score-assignment for age, we used the other formula defined in the methods to assign values to each of the other variables (Table 3).

The risk probability corresponding to each score was calculated using the formula: *p* = [1 + exp(*lp*)]^−1^. In this formula, the linear predictor (lp) was obtained by multiplying the value of each variable with its associated regression coefficient and summing all the values (*lp* = −∑_*i*=0_^*p*^*β*_*i*_*X*_*i*_). The results are shown as a nomogram (Figure 2).

## 4. Discussion

Venous thrombosis of the lower extremity is a well-known complication following lower limb fracture. Extensive research has been dedicated to the prevention and treatment of thrombosis, but early prediction of thrombosis is now appearing as an important research direction. In this paper, we analyzed clinical data of patients with lower extremity fractures from two centers from the past three years to develop a clinical prediction model for establishing the risk of DVT in such patients. The predictors used in this model are common and easily identified in clinical practice. Our final model showed strong predictive capability during the validation process (c − statistic = 0.676). This model will be effective in a clinical setting in the prediction of thrombosis in patients with lower extremity fractures. It is worth noting that the medical records of the thrombosis group and the nonthrombosis group are collected separately to compare the impact of each risk factor on thrombosis, so the number of medical records does not represent the incidence of thrombosis.

Numerous studies have been published on the prediction or screening of thrombosis in patients with lower extremity fractures or orthopedic surgery of the lower extremity. Some studies have evaluated the effect of a single factor on thrombosis. Monreal et al. collected the test results of 1033 patients undergoing large joint replacement surgery both at the time of discharge and during follow-up [20]. Using these clinical data, they assessed the efficacy of a combined strategy, that is, physical examination and compression ultrasound, to detect DVT prior to discharge. They found that a diagnostic testing for DVT before discharge has the capacity to identify 44% of patients who will experience symptoms after discharge. Madhav et al. conducted a retrospective analysis of 169 patients who were treated with open reduction and internal fixation for hip fractures and found that BMI is a significant predictive indicator of postoperative complications following an acetabular fracture [21]. Although the authors analyzed the impact of multiple factors on thrombosis, no clear scoring table or model was established. Rogers et al. conducted a cross-case study of 16,781 participants and found that factors predisposing to thrombosis included the following: infection, erythropoietin and blood transfusion, surgery, fracture, immobilization, and chemotherapy [22]. Park et al. performed a retrospective analysis of 901 lower limb fracture cases and identified several risk factors for increased DVT, including increased age, cardiovascular disease, and chronic lung disease [23]. Consequently, the predictive ability of some of the factors that we have identified as predictors has been verified in previous studies, verifying the validity of our results.

The article "Nomogram for Predicting Deep Venous Thrombosis in Lower Extremity Fractures" was retracted in 2024. Reasons: signs of a paper mill; suspected computer-generated content; unreliable results or conclusions; concerns about the data.

Overall, using a large multicenter sample, we analyzed multiple possible risk factors that have evident influence and have developed an easy-to-use model, which would be convenient for a clinical setting. Notably, in contrast with the Caprini score, our model includes energy at the time of impact and the type of surgical fixation of the fracture site, making our tool more specific for trauma patients with lower limb fractures. In addition, the risk factors included in the final model are well-defined and easy to be collected. Finally, calculating the final results through a score table or nomogram increases the practicality and accuracy of our model.

The limitations of this study should be acknowledged. First, as this is a retrospective study, issues with the patients' examination and treatment plans became apparent when collecting medical records. For example, in older records, doctors would only perform ultrasound test on patients with high thrombosis risk. Therefore, some patients without thrombosis or some patients with asymptomatic thrombosis did not undergo ultrasound testing during hospitalization. Since the thrombosis of these patients cannot be confirmed, such patients had to be excluded from the analysis. This reason may help explain why factors that are well-known predictors of thrombosis, such as D-dimer, were not included in our final model [8]. Therefore, this model may be more likely to be applied to a population at high risk of thrombosis, with a narrower scope than originally planned. Ideally, in future studies, we would seek to refine this model, by verifying the model in a clinical setting, as well as prospectively, comprehensively documenting case data and analyzing the correlation between factors which were not included in the model and DVT. Second, in this study, anticoagulation therapy for all patients was low-molecular-weight heparin sodium. However, anticoagulation drugs that are known to be effective and are clinically used include low-molecular-weight heparin, vitamin K antagonists, direct thrombin inhibitors, and direct FXa inhibitors [7, 9, 30]. Hence, in future studies, cases using different anticoagulation drugs should be included in the analysis for comparison. Moreover, although the risk factors included in the final model are simple and easy to complete, the addition of some inspection indicators and test results will improve the predictive ability of the model. For example, studies have shown that microRNA-495 and Stat3 proteins in the circulating blood can be used as biomarkers for the prognosis and prediction of lower extremity DVT [15]. Finally, our model was built using data from Wuhan, Hubei, and Shijiazhuang, Hebei, China, where all of the patients are Asian. Verification of our model in the white and black population is necessary.

The article "Nomogram for Predicting Deep Venous Thrombosis in Lower Extremity Fractures" was retracted in 2024. Reasons: signs of a paper mill; suspected computer-generated content; unreliable results or conclusions; concerns about the data.

## 5. Conclusion

Our study is the first, to the best of our knowledge, to provide a prediction model that can be used to guide decisions regarding primary prevention of venous thrombosis in patients with lower extremity fractures. During validation, the model showed good predictive ability. Our proposed score calculation method corresponding to the chart is designed to be convenient for clinical use. Overall, this model offers promising potential as a tool for the prevention and treatment of thrombosis in patients with lower limb fractures.

## Figures and Tables

**Figure 1:** Calibration curve of the clinical prediction model. On the calibration curve, *x*-axis is the nomogram predicted probability of thrombosis for low limb fracture patients, and *y*-axis is the actual probability of thrombosis for these patients.

**Figure 2:** Nomogram for the computation of percentage risk of lower extremity fracture-related thrombosis.

**Table 1:** Patients characteristics and univariate associations for thrombosis-related risk factors.

Risk factor	Thrombosis group (*n* = 1666)	Nonthrombosis group (*n* = 996)	*p* value
Sex [*n* (%)]			0.0018^#^
Male	870 (52.22%)	458 (45.98%)	
Female	796 (47.78%)	538 (54.02%)	
Age [median (IQR)]	73 (25.5)	64 (34)	<0.0001^@^
BMI [median (IQR)]	23.46 (4.72)	23.88 (4.89)	0.0023^@^
Fracture site [*n* (%)]			0.001^#^
Tibia/fibula	299 (17.95%)	88 (8.84%)	
Femur	1199 (71.97%)	835 (83.84%)	
Hip	168 (10.08%)	73 (7.33%)	
Energy [*n* (%)]			0.1085^#^
Low	1209 (72.57%)	751 (75.40%)	
High	457 (27.43%)	245 (24.60%)	
Open wound [*n* (%)]			0.0014^#^
No	1481 (88.90%)	923 (92.67%)	
Yes	185 (11.10%)	73 (7.33%)	
Traumatic brain injury [*n* (%)]			0.1611^#^
No	1553 (93.22%)	942 (94.58%)	
Yes	113 (6.78%)	54 (5.42%)	
Cardiovascular history [*n* (%)]			<0.0001^#^
No	1102 (66.15%)	579 (58.13%)	
Yes	564 (33.85%)	417 (41.87%)	
History of type II diabetes [*n* (%)]			0.0151^#^
No	1447 (86.85%)	831 (83.43%)	
Yes	219 (13.15%)	165 (16.57%)	
Smoking history [*n* (%)]			0.5171^#^
No	1482 (88.96%)	894 (89.76%)	
Yes	184 (11.04%)	102 (10.24%)	
Blood lipid [median (IQR)]			
TG	1.04 (0.72)	1.04 (0.67)	0.3573^@^
HDL	1.17 (0.5)	1.20 (0.44)	0.0971^@^
LDL	2.24 (0.95)	2.27 (0.92)	0.1570^@^
D-dimer [median (IQR)]	2.2 (3.82)	1.99 (3.14)	0.1570^@^
Clotting function [median (IQR)]			
TT	15.3 (2.8)	15.1 (2.4)	0.0209^@^
PT	12.4 (2.00)	12.1 (1.7)	<0.0001^@^
APTT	29.4 (6.3)	30.8 (7.9)	<0.0001^@^
FIB	3.6 (1.6)	3.6 (1.3)	0.4257^@^
Duration of surgery [median (IQR)]	2.0 (1.3)	2.0 (1.2)	0.3389^@^
Fracture fixation type [*n* (%)]			<0.0001^#^
Internal fixation	1266 (75.99%)	882 (88.55%)	
External fixation	117 (7.02%)	22 (2.21%)	
Other types	283 (16.99%)	92 (9.24%)	
Blood transfusion during hospitalization [*n* (%)]			<.0001^#^
No	879 (52.76%)	348 (34.94%)	
Yes	787 (47.24%)	648 (65.06%)	
Anticoagulation drugs [*n* (%)]			<0.0001^∗^
No	312 (18.73%)	42 (4.22%)	
Yes	1354 (81.27%)	954 (95.78%)	

^#^Comparison among groups using *χ*^2^ or CMH-*χ*^2^; ^∗^Comparison among groups using Fisher's exact probability test; ^@^Comparison among groups using the Wilcoxon rank-sum test; IQR: interquartile range.

The article "Nomogram for Predicting Deep Venous Thrombosis in Lower Extremity Fractures" was retracted in 2024. Reasons: signs of a paper mill; suspected computer-generated content; unreliable results or conclusions; concerns about the data.

**Table 2:** Multivariate logistic regression analysis.

Risk factor	Coef (*β*)	Wald-*χ*^2^	*p* value	OR	95% CI for OR
Intercept	-5.0642	-11.37	<.0001	—	—
Age	0.0192	7.16	<.0001	1.02	1.01-1.02
BMI	0.0484	4.05	<.0001	1.05	1.03-1.07
Energy	0.4054	3.51	0.0004	1.45	1.16-1.88
Fracture fixation type					
External fixation	Ref				
Other types	0.3807	1.38	0.1677	1.46	0.85-2.51
Internal fixation	0.9015	3.63	0.0003	2.46	1.51-4.01
Blood transfusion during hospitalization	0.3868	4.26	<.0001	1.47	1.23-1.76
Anticoagulation drugs	1.1537	6.49	<.0001	3.17	2.24-4.49

**Table 3:** Risk score chart for thrombosis in patients with lower extremity fractures.

Risk factor		Coef	Nomogram	Point
Age		0.0192	1.728	
	10			0
	20			10
	30			20
	40			30
	50			40
	60			50
	70			60
	80			70
	90			80
	100			90
	110			100
BMI		0.0484	2.45	
	10			0
	12			5
	14			10
	16			15
	18			20
	20			25
	22			29
	24			34
	26			39
	28			44
	30			49
	32			54
	34			59
	36			64
	38			69
	40			74
Fracture fixation type				
	External fixation	Ref	Ref	0
	Other types	0.3808	0.3808	20
	Internal fixation	0.9015	0.9015	52
Energy				
	Low	Ref	Ref	0
	High	0.4054	0.4054	23
Blood transfusion				
	No	Ref	Ref	0
	Yes	0.3868	0.3868	22
Anticoagulation drugs				
	Yes	Ref	Ref	0
	No	1.1537	1.1537	58

## Data Availability

If the original data is reasonably required, the permission to obtain can be applied to Professor Guohui Liu.
